# The Efficacy and Safety of Oral Nutrient Solution Supplementation in Patients with Esophageal Cancer under Nutritional, Psychological, Physical, and Prognostic Survival Differences

This article has been retracted.

**DOI:** 10.1155/2023/5055869

**Published:** 2023-02-09

**Authors:** Juntao Hao, Zengqiang Shen

**Affiliations:** Thoracic Surgery Department, Shanxi Provincial People's Hospital, Taiyuan, Shanxi 030012, China

## Abstract

Inflammasomes are massive intracellular multiprotein signaling complexes produced in the cytosolic compartment. Tumor etiology involves dysregulation of NLRP3 inflammasome activation. Current studies are being conducted to ascertain the effectiveness and safety of oral nutrient solution supplementation in patients with esophageal cancer based on the current understanding of the role of the NLRP3 inflammasome in possible cancer promotion and therapy. This study examines how oral nutrient solution supplement therapy affects patients receiving radiotherapy and chemotherapy for esophageal cancer in terms of nutrition, physical composition, quality of life, psychology, prognosis, and survival. A total of 120 patients with esophageal cancer admitted to our hospital from March 2020 to January 2021 were selected for the current study. The selected 120 patients are divided into nutritional supplement and traditional groups according to the random number table method, with 60 cases in each group. The nutritional supplement group received an oral nutritional solution, whereas the conventional group received the ordinary dietary intervention. Since radiotherapy can potentially damage healthy tissue with short- and long-term negative effects. Inflammatory reactions are a common component of adverse effects of early and late ionizing radiation. Oral nutrient solution supplement therapy for patients with esophageal cancer after radiotherapy and chemotherapy can significantly improve the levels of blood nutrients, later physical components, and quality of life of patients.

## 1. Introduction

Persistent infection and inflammation may play a role in developing different types of cancer in humans. Several inflammasomes, such as NLRP3, NLRP6, NLRC4, NLRP1, and AIM2, may harm cancer by modulating innate and adaptive immunity, apoptosis, differentiation, and the gut microbiome [1]. The quality of life esophageal cancer often occurs in the esophageal epithelium and is a malignant tumor of the digestive system. In addition, esophageal cancer frequently occurs in middle-aged and elderly patients, and its morbidity and mortality rank among all malignant tumor diseases, which seriously impact the human body and life [2]. Currently, radiation and chemotherapy are the go-to treatments for esophageal cancer. However, these treatments have some unfavorable side effects (radioactive esophagitis, esophageal bleeding, malnutrition, radioactive stomatitis, etc.), which can negatively impact patients' physical and mental health and quality of life. As a result, patients with esophageal cancer must receive specific nutrition support [3]. Several inflammasomes have been discovered, including NLRP1, NLRP2, NLRP3, missing in melanoma 2 (AIM2), and NLRC4. The NLRP3 inflammasome, a protein with a pyrin domain, is the one among them that is well described [4]. Cancer Nutrition Committee of The Chinese Anti-Cancer Society et al. [5] proposed in the nutritional treatment guidelines for patients with esophageal cancer that severe malnutrition should be first treated with nutritional intervention. Patients with mild or moderate malnutrition need to be given nutrition popularization, and nutritional intervention has not been determined. Studies have shown that dietary support following radiotherapy and chemotherapy can successfully prevent problems and enhance patients' quality of life [6]. Malignancies like colon cancer and melanoma are linked to NLRP3 inflammasome polymorphisms. They modify cell death, proliferation, gut microbiota, and innate and adaptive immunological responses, and NLRP1, NLRP3, NLRC4, NLRP6, and AIM2 impact cancer pathogenesis. While excessive inflammation caused by the inflammasome or the IL1 signaling pathways promotes breast cancer, fibrosarcoma, gastric carcinoma, and lung metastases in a context-dependent manner, it is mainly protective in colon cancer linked with colitis [7].

Inflammasomes can recognize endogenous danger signals as an inflammatory immune response. The NLR pyrin family domain containing 3 (NLRP3) inflammasome is the most prevalent and is linked to the development of many cancers. The role of the NLRP3 inflammasome in esophageal cancer (EC) has, however, only sometimes been discussed. According to the findings, the NLRP3 inflammasome is increased in human ESCC tissues, and this upregulation promotes the advancement of ESCC. NLRP3 may represent a viable new candidate for diagnostic and prognostic targets [8]. As a result of NLRP3's ability to respond to various inflammatory viral and endogenous ligands, including PAMPs and DAMPs, dysregulation in NLRP3 function is linked to the pathogenesis of a number of inflammatory diseases. Radiotherapy has both short- and long-term side effects and the potential to harm healthy tissue. Early and late ionizing radiation side effects frequently involve inflammatory responses [9]. However, there are currently limited clinical data and few investigations on oral nutritional solutions in patients receiving radiotherapy and chemotherapy for esophageal cancer to recover from the damage and side effects of radiotherapy and chemotherapy. Based on this, oral nutrient solution supplement therapy was used in this study for patients receiving radiotherapy and chemotherapy for esophageal cancer. It was discovered to help improve the patient's nutritional status and quality of life.

## 2. Method and Material

### 2.1. Sampling

A total of 120 patients with esophageal cancer identified and cured in the hospital from March 2020 to January 2021 were arbitrarily chosen and split into the nutritional supplement group and the traditional group according to the random number table method, with 60 cases in each group. The conventional group's age ranged from 60 to 81 years, with an average of 67.313.22 years, and the ratio was 27/33. The proportion of upper/middle/lower segment lesions was 29/11/20. In the nutritional supplement group, both were 25/35, aged from 61 to 80 years, with an average of 66.52 ± 4.13 years. The proportion of upper/middle/lower segment lesions was 27/12/21. All subjects' baseline data were comparable and did not reveal any statistically significant differences (*P* > 0.05).

Inclusion criteria are the following:

- Esophageal cancer was diagnosed according to clinicopathological examination results and diagnostic criteria
- No other malignant tumors
- Normal cognitive and behavioral functions
- No history of drug allergy
- Patients and their relatives signed informed consent in the case of clear study procedures

Exclusion criteria are the following:

- Combined with other diseases
- Heart, brain, liver, and kidney dysfunction
- Allergic to drugs in this study
- Patients with an expected survival period of fewer than 3 months

### 2.2. Procedure

Patients in the traditional group received routine diet nursing intervention, and medical staff reminded patients and their families to pay attention to postoperative diet, according to the hospital's own routine diet nursing program for dietary nursing. At the same time, during hospitalization, medical staff should regularly observe the body weight of patients, urge patients and their families to understand the knowledge of radiotherapy and chemotherapy, and know the prevention and alleviation of postoperative adverse reactions and complications; 1~3 months after discharge, medical staff should conduct regular telephone follow-up to understand the patient's physical and mental health and complications at the present stage.

Patients in the nutritional supplement group received healthy oral solutions from patients in the traditional group, and a nutritional support group was established. In order to facilitate discussions between nutritionists and nurses about patients' problems, our hospital's authoritative nutritional doctor was chosen as the group's leader. He sternly advised patients to take oral nutritional solutions following the recommended dosage. The nutrient solution (Xi'an Labon Clinical Nutrition Co., Ltd.) used in this study was composed of rishikang enteral nutrition formula food, including four preparations including 40 g rishikang homogenate dietary fiber type, 180 g rishikang whole protein nutritional liquid powder, 20 g rishikang vita, and 15 g dietary fiber. The nutritional ratio of the agent is 32.1 g sugar, 43.4 g protein, 36.5 g fat, 135 g carbohydrate, 25.3 g cellulose, including 1043 kcal, and 6.9 g nitrogen content. Protein : fat : carbohydrate heating ratio is 17 : 31 : 52. The nutritional solution chosen for this study includes high protein, high calorie, and high dietary fiber content. Each bottle contains 252 ml and 347 kcal, 3 bottles per day, and one bottle is drunk at an interval of about 5 h.

### 2.3. Observation Indicators

- Blood nutritional indexes of patients in the two groups were observed as follows: blood nutritional indicators were detected 1 week after surgery. 2 ml elbow venous blood was taken from the patient on a fasting stomach in the morning, stored at -40°C, and centrifugated for 5 min at 3000 r/min. Hemoglobin, plasma albumin, and plasma preprotein were detected and analyzed by an automatic biochemical analyzer (Hitachi 7180). Blood nutritional indexes (body weight, albumin, and prealbumin) were observed at admission, discharge, and 1 month and 3 months after discharge
- Observing two groups of patients with the changes of the physical components of the intervention, on the basis of InBodyS10 on two groups of patients on admission, 7 d after surgery, and 1 month after discharge, the examination of the physical components, the difference between the second and first measurement as an early physical composition change, the difference between the third and the second measurement as a late physical composition change. The patients in the two groups had their pertinent physical measurements taken, including body weight, fat-free body weight, basal metabolic rate, bone mineral content, body fat, body cells, muscle mass, and BMI [10]
- The negative emotions of patients in the two groups were observed before intervention, 1 month after intervention, and 3 months after intervention. The negative emotions of patients were assessed by self-rating anxiety scale (SAS) and depression rating scale (SDS). The higher the score was, the more serious the negative emotions of patients were
- Patients' quality of life (mental function, physical function, physical function, and social function) were scored according to QOLS before intervention, 1 month after intervention, and 3 months after intervention. The higher the score was, the higher the quality of life was
- Postoperative complications like anastomotic stenosis, severe diarrhea, reflux esophagitis, anastomotic fistula, and functional gastric emptying disorder were noted in the two groups after examining the incidence of complications in the two groups
- The survival of the subjects one year after treatment was followed up, and the Kaplan-Meier curves were drawn to analyze the survival rate of the subjects one year after birth

### 2.4. Statistical Methods

Software called SPSS26.0 was used to analyze the data. Measurement data were represented by the mean ± and standard deviation. For all groups, the *t*-test was utilised. All groups underwent the *x*^2^ test, which represents counting data as a percentage (percent). The *F* test was used to compare several datasets. The Mauchly test was performed to compare the data within the group at various times. The covariance matrix had a lot of football symmetry (*P* > 0.05), and the difference was statistically significant (*P* > 0.05).

## 3. Results

### 3.1. Changes of Blood Nutritional Indexes at Different Time Points

There was no significant difference in blood nutritional indexes between patients at admission and discharge (*P* > 0.05). The nutritional indexes 1 month after discharge and 3 months after discharge showed an increasing trend, and the indexes in the nutritional supplement group were higher, with statistical differences (*P* < 0.05) (see Table 1 and Figure 1).

### 3.2. Comparison of Physical Components between the Two Groups

There was no statistical difference in early constitution components of all subjects (*P* > 0.05). Body weight, body fat, and BMI all increased significantly and showed statistical differences (*P* < 0.05) in the late nutritional supplement group, as displayed in Table 2.

### 3.3. Changes of Negative Emotions at Different Time Points

The two negative mood indicators of the subjects showed a decreasing trend, and the decrease was greater in the nutritional supplement group, with statistical differences (*P* < 0.05) (see Table 3 and Figure 2.

### 3.4. Changes of QOLS Scores at Different Time Points

The scores of the 4 life quality dimensions of the study subjects showed an increasing trend, and the increase was greater in the nutritional supplement group, with statistical differences (*P* < 0.05) (see Table 4 and Figures 3 and 4.

### 3.5. Differences in the Occurrence of Long-Term Adverse Reactions

The incidence of anastomotic stenosis, severe diarrhea, functional gastric empting disorder, and anastomotic fistula was higher in the nutritional supplement group with statistical differences (*P* < 0.05) (Table 5).

### 3.6. Survival Analysis

The 1-year survival rate in the nutritional supplement group was significantly higher than that in the traditional group (*P* < 0.05) (see Figure 4).

## 4. Discussion

Esophageal cancer is one of the common malignant tumors in clinical practice, and its incidence is only lower than that of gastric cancer [11]. The pathogenesis of this disease has not been determined yet, Genetics and dietary habits, which have a significant impact on patients' physical and mental health as well as their quality of life, are thought to be associated to it [12]. At the present stage, radiotherapy and chemotherapy is the gold plan for the treatment of this disease, which has a certain effect on patients with esophageal cancer. Inflammatory reactions are a common component of both the early and late effects of radiation therapy. Due to the large variety of inflammatory infectious and endogenous ligands that NLRP3 responds to, including PAMPs and/or DAMPs, dysregulation in NLRP3 function is linked to the aetiology of many inflammatory disorders. However, patients with esophageal cancer are usually accompanied by malnutrition. If nutrients are not provided to patients in time after surgery, the nutritional status of patients after treatment will be poor, affecting the treatment effect. Therefore, nutritional care is essential for patients with esophageal cancer after radiotherapy and chemotherapy [13]. Exploring potential dietary changes may be utilised as therapeutic approaches to suppress Nlrp3 activation and the role of metabolites in controlling the activation of the canonical Nlrp3 inflammasome.

Patients with esophageal cancer are prone to body mass loss, anemia, and hypoproteinemia after radiotherapy and chemotherapy, leading to a significant decline in blood nutritional indicators [14]. According to [15] by building model of nutrition support in patients with esophageal cancer radiotherapy launched to explore the influence of nutritional status and quality of life, it was found that two groups of patients at the time of admission and discharge of blood nutrition index have no obvious change, but in 1 month to 3 months after hospital discharge blood nutritional indexes, obvious rising trend was observed, and the results are consistent. In this study, 1-3 months after discharge, body weight, albumin, and prealbumin indexes significantly increased in both the nutritional supplement group and the traditional group, the nutritional supplement group showing more pronounced growing trend. According to an analysis of the process, oral nutrient solutions with high protein and high dietary fiber content can maintain patients' nutritional status and enhance their blood nutritional indicators.

Siguang and Strong Yong [16] found in the study that the difference in early physical composition between the two groups was mainly in the muscle and water in lower limbs, while other physical composition remained unchanged. Body composition changes in the later time were primarily related to changes in body weight, fat-free body weight, and muscle mass, which were unrelated to this study. This study showed that there was no significant difference in the changes of early constitution components between the two groups. However, the body weight, body fat, and BMI of patients in the latter group were significantly higher than those in the traditional group. The mechanism may be that the sugar, protein, fat, and other components in the nutrient solution are conducive to the increase of patients' body weight and body fat, and the nutrient solution is liquid food, which can be better absorbed by patients and help to supplement the loss of patients' constitution components after surgery. Domestic scholar Shuang [17] found that SAS and SDS scores were significantly reduced after intervention. Wang et al. [18] found that vitamin D supplementation can significantly reduce the adverse mood of patients. The above conclusions are consistent with the results of this study. As per [19], various dietary interventions have been explored that may have an effect on sterile inflammatory illness and emphasise the importance of energy substrates, alternative fuels, and metabolic DAMPs in the regulation of the NLRP3 inflammasome. Combined with SAS, SDS score data analysis of this study found that the supplement group's negative emotions have significantly lower score than that of the traditional group, which further illustrate that esophageal cancer can cause great pressure to the patients' psychological, lead to bad feelings, and affect patients' physical and mental health; the patient oral solution can make patients feel valued and further increase the patients confidence. It can obviously reduce the patient's physical and mental pressure and relieve the bad mood. According to the findings, thymoquinone therapy in a mouse model reduced metastatic melanoma by downregulating NLRP3 and reducing IL-1 and IL18 release.

Patients with esophageal cancer will have obvious adverse reactions after radiotherapy and chemotherapy, which seriously affect the physical health and quality of life of patients. After radiotherapy and chemotherapy, nutritional supplementation can greatly enhance this scenario [20]. According to Qian et al. [21], patients who got nutritional supplementation scored higher after intervention, proving that more sophisticated nutritional support can enhance patients' quality of life. According to Chaoyang [22], nutritional support for esophageal cancer patients can greatly enhance their nutritional status and quality of life. Preoperative nutritional supplementation has been found in several trials to dramatically lower the incidence of postoperative problems and enhance patients' nutritional condition [23]. The NLRP3 inflammasome's role in cancer progression in vivo is yet unknown and has to be confirmed. It has been proposed that the tissue environment particularly determines whether cancer is inhibited or stimulated when inflammasomes are activated [10]. Because NLRP3 responds to a variety of inflammatory infectious and endogenous ligands, including PAMPs and/or DAMPs, dysregulation in NLRP3 function is linked to the aetiology of a number of inflammatory diseases. The results of this study showed that QOLS score increased more significantly in patients who received oral nutrient solution. Oral nutrient solution contains a large amount of protein, carbohydrates, and dietary fiber and a high-quality liquid diet, which is an effective nutritional support for patients and can significantly improve the quality of life of patients. At the same time, oral nutrient solution contains a large amount of dietary fiber, which can improve stomach function, accelerate stomach peristalsis, and further reduce postoperative complications.

## 5. Conclusion

Based on the current knowledge of the impact of the NLRP3 inflammasome on potential cancer promotion and therapy, studies are currently being done to determine the efficacy and safety of oral nutritional solution supplementation in patients with esophageal cancer. The identification of the NLRP3 inflammasome's function in various tumor types is receiving more attention. However, there is still debate and contradicting evidence regarding the involvement of inflammasomes in tumor development and invasion. Radiation therapy can potentially injure healthy tissue and has both short- and long-term negative effects. However, there are currently few studies and scant clinical data on oral nutritional supplements in esophageal cancer patients receiving radiation and chemotherapy to repair the harm and side effects of radiation and chemotherapy. The results show that the blood nutritional indexes showed an increasing trend 1-3 months after discharge, and the range of changes was larger in the nutritional supplement group (*P* < 0.05). The body weight, body fat, and BMI in the nutritional supplement group were significantly higher than those in the traditional group (*P* < 0.05). The negative emotions showed a decreasing trend, and the decreasing range was greater in the nutritional supplement group (*P* < 0.05). Similarly, the QOLS score showed an increasing trend, and the range of change was larger in the nutritional supplement group (*P* < 0.05). The incidence of adverse reactions in the nutritional supplement group was significantly lower than that in the traditional group, and the 1-year survival rate was higher (*P* < 0.05). Hence, oral nutrient solution supplement therapy for patients with esophageal cancer can significantly increase blood nutrient levels. Omega-3 fatty acid supplementation has promising characteristic of reducing the pathogenic effects of metabolite-stimulated Nlrp3. However, there are still some defects in this study. To establish a more solid foundation for postoperative nutritional treatment for patients with esophageal cancer, additional research with a bigger sample size is required.

## Figures and Tables

**Figure 1:** Changes of blood nutritional indexes at different time points. Note: A, B, C, and D represent compared with other time points, *P* < 0.05; # represents the comparison with the traditional group, *P* < 0.05.

**Figure 2:** Changes of negative emotions at various places. Note: denotes the comparison with the usual group, *P* < 0.05, and A, B, and C represent *P* > 0.05 compared with various time points.

**Figure 3:** Changes of QOLS scores at different time points. Note: same as Figure 2.

**Figure 4:** Difference in 1-year survival rate.

**Table 1:** Changes of blood nutritional indexes at different time points ($\bar{x}\pm s$, *n* = 60).

Group	Time point	Body quality (kg)	Albumin (mg/L)	Prealbumin (mg/L)
Nutritional supplement group (*n* = 60)	On admission	57.24 ± 6.12	35.27 ± 3.11	16.87 ± 5.21
	When discharged from hospital	58.71 ± 6.91	37.24 ± 4.01	19.22 ± 5.95
	She was discharged for 1 month	64.21 ± 6.01	45.72 ± 3.49	21.85 ± 5.33
	He was discharged for 3 months	65.19 ± 6.31	52.35 ± 3.92	26.64 ± 5.03

Traditional group (*n* = 60)	on admission	57.02 ± 5.89	35.87 ± 3.08	16.38 ± 5.17
	When discharged from hospital	58.79 ± 5.88	36.88 ± 3.98	18.98 ± 6.04
	She was discharged for 1 month	59.07 ± 5.22	39.49 ± 4.16	19.65 ± 5.23
	He was discharged for 3 months	59.63 ± 6.04	44.76 ± 4.29	22.33 ± 4.78

*F*_Time point_		434.322	412.212	403.042

*P*_Time point_		<0.001	<0.001	<0.001

*F*_Time point∗group_		413.332	409.212	455.022

*P*_Time point∗group_		<0.001	<0.001	<0.001

**Table 2:** Comparison of constitution components between the two groups $\left(\bar{x}\pm s\right)$.

Project	Early physical composition changes			Later physical composition changes		
	Traditional group	Nutritional supplement group	*P*	Traditional group	Nutritional supplement group	*P*
Weight (kg)	−0.12 ± 1.57	0.06 ± 1.37	0.341	−4.23 ± 1.66	−1.37 ± 2.67	0.001
Fat-free body weight (kg)	0.01 ± 3.27	0.13 ± 3.71	0.872	−5.22 ± 3.12	−4.89 ± 3.15	0.057
Body fat (kg)	−0.24 ± 3.01	−0.13 ± 3.47	0.624	0.87 ± 3.79	2.37 ± 3.11	0.001
Muscle mass (kg)	0.18 ± 3.76	−0.01 ± 3.17	0.698	−5.33 ± 3.28	−3.77 ± 3.17	0.031
BMI (kg/m^2^)	−0.09 ± 0.72	0.01 ± 0.62	0.377	−1.78 ± 0.76	−0.23 ± 1.01	0.001
Basal metabolic rate (kcal)	−21.79 ± 179.24	2.33 ± 71.34	0.392	−89.22 ± 165.34	−82.65 ± 62.77	0.765
Body cell volume (kg)	−0.07 ± 1.89	−0.01 ± 1.99	0.881	−3.47 ± 2.55	−2.98 ± 2.31	0.117
Bone mineral content (kg)	0.09 ± 0.41	0.13 ± 0.41	0.831	−0.39 ± 0.41	−0.39 ± 0.41	0.434

**Table 3:** Changes of negative emotions at different time points (*n* = 60$\left(\bar{x}\pm s\right)$).

Group	Time point	SAS	SDS
Nutritional supplement group	Before the intervention	59.77 ± 4.23	58.37 ± 4.97
	One month after the intervention	41.33 ± 3.23	48.41 ± 4.27
	Three months after the intervention	32.91 ± 4.21	33.61 ± 5.12

Traditional group	Before the intervention	59.48 ± 4.57	61.31 ± 4.78
	One month after the intervention	51.91 ± 4.61	53.67 ± 5.21
	Three months after the intervention	42.91 ± 4.61	43.67 ± 5.21

*F*_Time point_		412.102	411.202

*P*_Time point_		<0.001	<0.001

*F*_Time point∗group_		401.212	402.012

*P*_Time point∗group_		<0.001	<0.001

**Table 4:** Changes of QOLS scores at different time points $\left(\bar{x}\pm s\right)$.

Group	Time point	Social function	Physiologic function	Physical function	Mental function
Nutritional supplement group	Before the intervention	60.66 ± 9.87	67.88 ± 11.12	58.98 ± 10.78	51.64 ± 7.56
	One month after the intervention	70.16 ± 11.08	77.38 ± 11.10	68.48 ± 10.65	61.14 ± 8.23
	Three months after the intervention	79.07 ± 12.89	86.43 ± 11.09	78.70 ± 10.57	71.76 ± 8.67

Traditional group	Before the intervention				
	One month after the intervention	58.77 ± 9.32	68.50 ± 10.76	56.81 ± 10.65	51.69 ± 7.77
	Three months after the intervention	64.27 ± 10.13	74.00 ± 10.54	62.31 ± 10.45	59.19 ± 7.82
	Time point	69.91 ± 11.97	78.50 ± 10.13	66.81 ± 9.89	63.69 ± 7.79

*F*_Time point_		416.542	421.532	432.543	444.521

*P*_Time point_		<0.001	<0.001	<0.001	<0.001

*F*_Time point∗group_		534.324	526.308	514.231	521.312

*P*_Time point∗group_		<0.001	<0.001	<0.001	<0.001

**Table 5:** Differences in the occurrence of long-term adverse reactions (*n* = 60 (%)).

Group	*N*	The anastomosis is narrow	Reflux esophagitis	Severe diarrhea	Functional gastric emptying disorder	Anastomotic fistula
Nutritional supplement group	60	2 (3.33)	3 (5.00)	2 (3.33)	1 (1.67)	2 (3.33)
Traditional group	60	12 (20.00)	4 (6.67)	6 (10.00)	5 (8.33)	8 (13.33)
*x* ^2^	5.341	4.273	0.223	5.221	4.768	5.314
*P*	0.001	0.001	0.546	0.001	0.001	0.001

## Data Availability

The dataset used in this paper are available from the corresponding author upon request.
